# Application of Virtual Reality Based on 3D-CTA in Intracranial Aneurysm Surgery

This article has been retracted.

**DOI:** 10.1155/2021/9913949

**Published:** 2021-05-29

**Authors:** Zhilei Li, Guojin Huo, Yi Feng, Zhulin Ma

**Affiliations:** Department of Neurosurgery, The First Hospital of Yulin, Yulin 719000, Shaanxi, China

## Abstract

As a popular technology in the field of human-computer interaction, virtual reality (VR) brings a brand new sensory experience to users by generating the environment. In recent years, while introducing the application of virtual reality technology, researchers have done a lot of work around virtual reality in many fields, such as the application of virtual reality technology in medical procedures. Combining the immersive and expandable features of virtual reality can improve the safety and accuracy of surgery. This article mainly introduces the application of 3D-CTA virtual reality technology in intracranial aneurysm surgery and aims to provide some ideas and directions for the improvement and progress of intracranial aneurysm surgery. This paper presents a research method based on virtual reality technology 3D-CTA in intracranial aneurysm surgery, including the application overview of 3D-CTA in intracranial aneurysm surgery and the virtual reality algorithm based on 3D-CTA for intracranial arteries. In addition, there is also the application of virtual reality CTA technology in the design of the intracranial aneurysm application system. Experimental results show that the average accuracy of 3D-CTA diagnosis based on virtual reality is 90.81%, and it can be put into use in the next step.

## 1. Introduction

Intracranial aneurysm (IA) refers to the abnormal expansion of the walls of cerebral arteries, forming tumors similar to protrusions. This is a general cerebrovascular disease and the most common subarachnoid hemorrhage (SAH). Now, the incidence of intracranial aneurysms is increasing year by year, and the third category is cerebrovascular disorders, followed by ischemic stroke and hypertensive intracerebral hemorrhage (HICH). Once an intracranial aneurysm ruptures and hemorrhages, the prognosis is often poor. About 1/3 of the patients have died when they can be treated in the hospital in the future, 1/3 of the patients died in the hospital, and the other 1/3 of the patients received active treatment. Among them, the fatality rate of the aneurysm after rupture and bleeding can be as high as 60% to 80%. With the transformation of medical models and traditional medical concepts, neurosurgery has changed from simply treating the disease itself to maximizing the removal of the disease while reducing the impact of surgery on nerve function. Therefore, neurosurgery operations are required to be as simple and precise as possible, and it is a personalized treatment strategy that is reflected in each patient, and the three-dimensional visualization technology of medical images has emerged at the historic moment. The simple summary of the three-dimensional visualization of medical images refers to the three-dimensional reconstruction of the original series of images after the conversion, segmentation, registration, and fusion of the two-dimensional tomographic images obtained from CT, MRI, or ultrasound.

With the rapid and continuous development of science and technology, virtual reality technology gradually tends to mature and perfect and is widely used in various fields. At present, virtual reality technology has touched on large-scale exhibition activities and has become another effective form of exhibition activities. Virtual reality is an interdisciplinary comprehensive technology widely used in military, film, medical, gambling, and other fields. Virtual reality can simulate the objective world, visualize it, and make people feel trapped. Virtual surgery provides surgeons with a reusable surgical training platform and can help doctors perform preoperative rehearsals and prediction of surgical results, which is convenient to avoid risks. In addition, a simple surgical training device is provided, which provides a basis for the addition of materials and increases the operator's immersion in the virtual operating system. Virtual reality technology plays a very important role in the diagnosis and treatment of neurosurgical diseases, bringing medical care into a new era.

The Kitano study believes that there are many changes in the branching and operation of the pulmonary artery (PA) and pulmonary vein (PV). It is ideal to separate them as a surgical simulation of lung cancer, and it is important to perform video-assisted thoracoscopic surgery (VATS) before proceeding and to perform surgery quickly and safely. Therefore, Kitano evaluated the objective and subjective image quality of PA and PV of the split single-phase protocol (SBSPP) in preoperative three-dimensional computed tomography angiography (3D-CTA), including contrast attenuation, separation ability, and vessel visualization. Kitano sets the subjective image quality visualization of PA and PV until the level of segmentation is exceeded. At this time, SBSPP can obtain enough CT values to display PA and PV, respectively, and useful PA and PV 3D-CTA imaging before VATS. This method is more complicated and is not conducive to popularization in practice [1]. Fujioka found that portraying small blood vessels can provide doctors with useful preoperative information. Although angiography can visualize blood vessels in detail, it is invasive. MR angiography is a minimally invasive method of depicting blood vessels, but the image resolution is not sufficient for preoperative evaluation. In this study, Fujioka used a less invasive three-dimensional CT angiography (3D-CTA) and reconstructed an adaptive iterative dose resolution 3D (AIDR 3D) image with a display field of view (D-FOV). The image is suitable for large and wide arteries with small diameters and creates a fusion image. Compared with angiography, the created image allows observation of blood vessel branches in a large area and is less invasive. In addition, Fujioka evaluated the utility of 3D-CTA to visualize arterial branches and capillaries as a preoperative evaluation of tumor resection. This research lacks experimental data support and is not scientific [2]. In his research, Chen showed the latest developments in the omnidirectional video processing flow, including projection and evaluation. Unlike traditional video, omnidirectional video (also called panoramic video or 360-degree video) is in a spherical range, so special virtual reality technology tools are required. For this type of video, each picture should be projected onto a two-dimensional plane for encoding and decoding to adapt to the input of the existing video encoding system. Therefore, the coding impact of the projection and the accuracy of the evaluation method are very important in this pipeline. Chen introduced and classified the latest research developments, such as different projection methods that are beneficial to video coding, dedicated video quality evaluation indicators, and optimized transmission methods, etc., also stipulated the coding performance under different projection methods, and discussed omnidirectional video dealing with future trends. This research is one-sided and not practical [3, 4].

The innovations of this paper are as follows: (1) it designed an application system based on 3D-CTA virtual reality technology in intracranial aneurysm surgery; (2) it proposed head posture tracking technology to establish a system recognition and tracking module.

## 2. Application Research Method Based on 3D-CTA Virtual Reality Technology in Intracranial Aneurysm Surgery

### 2.1. Application of 3D-CTA in Intracranial Aneurysm Surgery

#### 2.1.1. Overview of Intracranial Aneurysms

Intracranial aneurysms are cerebral vasodilation caused by abnormal changes in local blood vessels. It may be caused by related or acquired causes such as trauma, inflammation, and high blood pressure. The first cause of subarachnoid hemorrhage (SAH) caused by spontaneous bleeding is about 54% to 75% [5]. Intracranial aneurysms mainly occur in middle-aged people between 40 and 60 years of age. This is a common stroke, second only to cerebral thrombosis and long-term cerebral hemorrhage. Most aneurysms are hidden before rupture and have no symptoms. Once they rupture and bleed, they are likely to close or even die [6, 7].

#### 2.1.2. 3D-CTA Treatment

DSA is the most valuable method for diagnosing aneurysms. It can specify the location, shape, size, direction, the number of aneurysms, and the relationship with the surrounding blood vessels. It can be used for intravascular surgery, but it has many traumas, long inspection time, and many complications and other problems.

At present, some noninvasive vascular imaging methods such as CT angiography (CTA) and MR angiography (MRA) have been widely used in the clinical diagnosis of cerebrovascular diseases. MRA is noninvasive and convenient with no radiation and no complications of cerebral angiography. It can show the brain parenchyma, understands the relationship between the aneurysm and brain tissue, and is not affected by skull artifacts [8]. However, MRA does not clearly display the arteries at the base of the skull and the peripheral segments. It has low sensitivity to aneurysms in these parts and takes longer than CTA. Patients with ruptured aneurysms are prone to artifacts due to agitation during the examination, which is not suitable for the examination of critically ill patients and patients who cannot cooperate with agitation. Since the MRA examination needs to be carried out in a strong magnetic field, the use of MRA in patients with metal implants such as pacemakers is limited [9, 10].

CTA has developed rapidly in recent years. Its radiation dose is smaller than DSA, and it is a noninvasive examination. Therefore, it is safer than DSA. It has a better display effect on blood vessels adjacent to bone structures such as the base of the skull. The CTA principle and operation are simple, the inspection time is short, the cost is low, and it has a good time and space resolution [11]. With the development of CT technology, especially the emergence of multislice spiral CT, and the rapid development of CTA three-dimensional image postprocessing technology, three-dimensional CT angiography (3D-CTA) has greatly improved the diagnostic ability of aneurysms [12]. The schematic diagram of intracranial three-dimensional CT angiography is shown in Figure 1 (due to the limited data source in this article, the picture comes from baidu.com).

#### 2.1.3. Treatment Steps

Patients diagnosed with spontaneous subarachnoid hemorrhage by CT should undergo CTA examination at an appropriate time. Patients who found intracranial aneurysms were directly treated by microsurgery according to the information provided by 3D-CTA. Those who did not find intracranial aneurysms were directly treated by microsurgery for the aneurysm and repeated imaging examinations by DSA-CTA. They compare and analyze the 3D-CIA image information with the image information and DSA image observed during the operation [13].

All patients used 16 spiral CT to check the speed of light. CTA adopts the advantage 9.0 software system, 220 V voltage, 120 mA current, scanning layer thickness of 0425 mm, the pitch of 0413 : 1, no reconstruction layer thickness, the total number of scanning layers of 70∼85, high-pressure syringe through anterior intravenous injection, a relative factor that is nonionic contrast factor Uweixin has with an injection rate of 3 ml per second, a total contrast factor of 60 ml, and a delay time of 14 to 21 seconds. Three-dimensional imaging processing methods are surface coating screen, maximum density display, volume reproduction, etc., of which the volume reproduction method is the most commonly used [14, 15].

### 2.2. Virtual Reality-Related Algorithms Based on Intracranial Aneurysm Surgery

#### 2.2.1. Signal Preprocessing Algorithm

Through the communication packet capture tool to capture the data sent by the VR surgery scene, through analysis, it is found that the data packets sent by the VR surgery scene form a first-order step system in each cycle [16]. According to the relevant principles of automatic cybernetics, the mathematical model of the first-order system can exactly represent it correctly [17]. The formula of the transfer function of the first-order system model is as follows, where *g* represents the input signal, *ϕ*(g) represents the output signal, and *t* is the time constant:

(1) $$\begin{array}{c} \phi \left(g\right)=\frac{1}{tg}+1. \end{array}$$

If the first-order transfer function can describe the model correctly, how to find the appropriate parameter T value becomes the key to solving the problem, which is related to the geometric meaning of the first-order transfer function [18]. Assuming that the unit step function *r*(*x*)=*p*(*x*) is input, the response function of the unit step can be obtained according to formula (1):

(2) $$\begin{array}{c} h\left(x\right)=p+e^{-x/t},\;x\geq 0. \end{array}$$

The transfer function is

(3) $$\begin{array}{c} \phi \left(g\right)=\frac{1}{5g}+1. \end{array}$$

Since the computer system is a discrete system, the continuous step function mentioned above cannot be directly recognized by the computer, so the continuous function needs to be discretized [19]. First, the transfer function is Z-transformed; then after the inverse transformation is performed, it is projected to the n-plane for n-transformation; finally, the difference equation is calculated and sorted out [20]. Define *k*(*g*) as a generalized continuous object and *k*(*z*) as a generalized discrete object; then, its generalized object pulse transfer function satisfies

(4) $$\begin{array}{c} k\left(z\right)=f\left[\frac{p-e^{gt}}{g}k\left(g\right)\right]. \end{array}$$

Then, we use the heuristic method to determine the structure of the controller *k*(*z*). The commonly used first-order form with phase lead and phase lag can be expressed as a pulse transfer function:

(5) $$\begin{array}{c} d\left(z\right)=k_{c}\frac{z-z_{c}}{z-p_{c}}. \end{array}$$

In formula (5), *z*_*c*_ represents the real zero point, and *p*_*c*_ represents the real pole in the unit circle. Since the analog controller cannot affect the steady-state performance of the system, there is a constraint *d*(*z*)*|*_*z*=1_=1. At this time, *k*_*c*_ is

(6) $$\begin{array}{c} k_{c}=\frac{1-p_{c}}{1-z_{c}}. \end{array}$$

*Z*-transform the transfer function

(7) $$\begin{array}{c} k\left(z\right)=f\left[\frac{p-e^{-gt}}{g}\times \frac{a}{g+a}\right]=\frac{1-e^{-at}}{z+e^{-at}}. \end{array}$$

Get the difference equation

(8) $$\begin{array}{c} c\left(k+1\right)=c\left(k\right)+T\left[-\frac{L-e^{-aT}}{T}c\left(k\right)+\frac{1-e^{-aT}}{T}u\left(k\right)\right]. \end{array}$$

Among them, *u*(*k*) is the input signal, *c*(*k*) is the output signal, and formula (8) represents the recurrence relationship between two adjacent cycles [21, 22].

#### 2.2.2. Force Feedback Algorithm

(1) Through the analysis of the dynamic equation of the spring-mass point model, the moving mass point satisfies the following differential equation:
  (9) $$\begin{array}{c} W\frac{\partial^{2}z}{\partial t^{2}}+D\frac{\partial z}{\partial t}+E_{\left(z\right)}z=f\left(z\right). \end{array}$$
Among them, *W* represents the mass of the mass point, *D* is the damping coefficient, *z* is the space coordinate of the mass point, *E* is the elastic coefficient of the spring, and *t* is the time constant [23]. The solution of the system equations can be transformed into the problem of solving the differential equations of discrete particles, and the approximate solution that satisfies the accuracy range is calculated [24]. If there is a unique solution to this equation, and Δ*t* is set as the unit time quantity, in any time period, through the time difference method and the increment method, for each discrete mass point, the differential equation can be transformed into
  (10) $$\begin{array}{c} m^{i}\frac{\partial^{2}z^{i}}{\partial t^{2}}=m^{i}\frac{1}{\Delta t^{2}}\left(z_{i+\Delta t}+z_{i}+z_{i-\Delta t}\right), \end{array}$$
  (11) $$\begin{array}{c} d\frac{\partial z^{i}}{\partial t}=d\frac{1}{\Delta t}\left(z_{t+\Delta t}-z_{t-\Delta t}\right), \end{array}$$
where *m*^*i*^ represents the quality of the i-th mass point, and *z*^*i*^ is the coordinate position of the *i*-th mass point. Substituting formulas (10) and (11) into formula (9), we get
  (12) $$\begin{array}{c} m^{i}\frac{1}{\Delta t^{2}}\left(z_{t+\Delta t}-z_{i}+z_{t-\Delta t}\right)+d\frac{1}{\Delta t}\left(z_{t+\Delta t}-z_{t-\Delta t}\right)\\ =f_{\text{ext}}^{i}\left(z_{i+\Delta t}\right)-f_{k}^{i}\left(z_{i+\Delta t}\right). \end{array}$$
When Δ*t* approaches infinity, *f*_ext_^*i*^(*z*_*i*+Δ*t*_) can be replaced with *f*_ext_^*i*^(*z*_*i*_), and *f*_*k*_^*i*^(*z*_*i*+Δ*t*_) can be replaced with *f*_*k*_^*i*^(*z*_*i*_), you can get
  (13) $$\begin{array}{c} \left(m^{i}\frac{1}{\Delta t^{2}}+d\frac{1}{\Delta t}\right)z_{t+\Delta t}=f_{\text{ext}}^{i}\left(z_{i}\right)-f_{k}^{i}\left(z_{i}\right)+m^{i}\frac{2}{\Delta t^{2}}z_{i}\\ -\left(m^{i}\frac{1}{\Delta t^{2}}+d\frac{1}{\Delta t}\right)z_{i-\Delta t}. \end{array}$$
(2) Among the force feedback algorithms, one representative method is Euler's method. The basic idea of Euler's method is to use the form of forward difference quotient to approximate the reciprocal and to discretize and solve the dynamic differential equation [25, 26], because there is the following formula in the mass point *m*^*i*^:
  (14) $$\begin{array}{c} z^{\prime }\left(m^{i}\right)=f\left(z^{i},f_{\text{ext}}^{i}\right),\;i=1,2,3,\ldots ,n. \end{array}$$

After approximating the derivative in the form of the forward difference quotient, we can get

(15) $$\begin{array}{c} \frac{z\left(m^{i}\right)-z\left(m^{i}\right)}{2\Delta t}=f\left(z^{i},f_{\text{ext}}^{i}\right), \end{array}$$

where Δ*t* is the unit time; when *t*=(*n* − 1)Δ*t*, the Euler integral formula is obtained; that is, the displacement is

(16) $$\begin{array}{c} z_{n-1}^{i}=z_{n}^{i}+\Delta tf\left(z^{i},f_{\text{ext}}^{i}\right). \end{array}$$

The method part of this article uses the above method to study the application of 3D-CTA virtual reality technology in intracranial aneurysm surgery. The specific process is shown in Figure 2 [25, 26].

## 3. Application System Design Based on 3D-CTA Virtual Reality Technology in Intracranial Aneurysm Surgery

### 3.1. Overall Design of the System

*Development Tools.* The development of the system is firstly modeling, and after the model is made, it is imported into the Unity3D platform to build the environment scene [27, 28]. Then, we complete the functions that the system needs to achieve by writing scripts. The main modules implemented by the system include UI display, simulating the CT scanning process, displaying CT scanning results, CT internal structure principles, and theoretical assessment. After the module function is realized, it can be published on the PC or Web, and the user can enter the designated webpage for learning. At the same time, the system can also be combined with HTC VIVE equipment to perform VR human-computer interaction to enhance the user's operating somatosensory. There are two tools required for system development, namely, modeling software and virtual reality development software. Among them, three-dimensional modeling software includes 3D Slash, Auto CAD, Maya, Mesh mixer, 3DS Max, and Inventor, and virtual reality development software includes Turn tool, Unity3D, Utility Toolkit, and VT [29]. Both 3D modeling and system development software have their focus. For example, some of the 3D modeling software is suitable for the modeling of characters, some are suitable for the establishment of architectural models, and some focus on the establishment of equipment models [30]. Virtual reality development software is also the same, some are suitable for system development, and some can simplify game development. According to the different characteristics and needs of these development tools, the tools suitable for the development of the system are selected.

### 3.2. Head Posture Tracking Technology

#### 3.2.1. VTK Coordinate System

VTK (Visualization Development Toolkit) is a tool for the study of graphical modeling of virtual operating systems in this article. VTK is mainly composed of four coordinate systems: model, world, view, and screen. The global coordinate system is the coordinate system where the participant is located, that is, the coordinate system where the virtual simulated surgical model is located. The coordinates and angle transformations of the machine model studied in this paper are all obtained by transformations related to this coordinate system. The projected coordinate system (camera coordinate system) is the coordinate system used to observe the experimental object. In research, it is necessary to observe experimental objects from various angles or distances [9, 10, 31].

#### 3.2.2. Method of Obtaining Head Posture

The PATRIOT device transmitter is installed on the upper middle of the user's forehead, so that the signal from the transmitter can better simulate personal visual contact. The PATRIOT receiver is placed directly behind the screen, and the operator's posture data is programmed to obtain the Developer Interface (PDI) provided by the PATRIOT device by using the Polhemus application program interface. This study uses the BO-OL ReadSinglePnoBuf provided by it. The first parameter of the function is the PBYTE type indicator, which is used to display the size of the storage unit receiver that stores the data of the frame obtained from it and the size of the second parameter storage unit. According to the above coding form, this article can obtain the position coordinates and position angle of the virtual doctor's head.

#### 3.2.3. Display under Threshold Control

After obtaining the three-dimensional coordinate data of the monitoring device, the established intracranial three-dimensional model is combined with the monitoring device. Because the coordinate data is constantly moving up and down in a small range, when the image and the tracking device are connected, the three-dimensional medical intracranial image we made will vibrate. In order to avoid this situation, we set a threshold to determine the real-time image whether the coordinates and angles change with the change of the head posture. At the same time, the threshold setting can also improve the response speed of the system and reduce the frequency of image reconstruction [32–34]. We know that each image reconstruction will take up a lot of system memory, and sometimes, the slight shift of the head is not to change the perspective or rotate the image. The establishment of the threshold helps the investigation to avoid irregular reconstruction, reduces the interference of unconscious patient behavior on image conversion and head position monitoring, and also increases the effective frequency of concealed reconstruction of images of human organs.

This part of the experiment proposes that the above steps are used to design an application system based on 3D-CTA virtual reality technology in intracranial aneurysm surgery. The specific process is shown in Table 1.

## 4. Based on 3D-CTA Virtual Reality Technology in Intracranial Aneurysm Surgery Application Research Analysis

### 4.1. Experimental Results and Analysis

1. In order to verify the superiority of the improved Euler algorithm used in the force feedback algorithm in the virtual reality system in this paper, the single-step execution time of the traditional Euler algorithm, the improved Euler algorithm, and the Runge-Kutta algorithm are now compared. A total of six experiments were carried out, and the results are shown in Table 2 and Figure 3.
2. It can be seen from the chart that among the three numerical calculation methods of the improved Euler algorithm, the traditional Euler algorithm, and the Runge-Kutta algorithm, the improved Euler method has the shortest single-step execution time and the fastest deformation frame rate. The evaluation of the effect of virtual surgery simulation includes three aspects: visual fidelity, tactile fidelity, and real time. The improved Euler method is adopted, the execution time is short, and the calculation efficiency is high, which fully meets the requirements of virtual surgery simulation [35].
3. The overall diagnosis of aneurysms was analyzed based on virtual reality CTA and DSA; based on intraoperative findings combined with DSA and 3D-CTA examination results, the aneurysms are divided into three groups according to the largest diameter: small aneurysm group (largest diameter <5 mm), middle aneurysm group (5 mm < maximum diameter <15 mm), and large aneurysm group (maximum diameter >15 mm). The diagnosis of aneurysms of different sizes was analyzed by CTA and DSA; the display of CTA and DSA was analyzed on the aneurysm body, tumor neck, tumor-bearing artery, and the anatomical structure of the operation area. The basis for the final diagnosis of aneurysm is as follows: the final diagnosis is the result of intraoperative exploration in the case of surgical treatment, and the result of DSA in the case of no surgical treatment. Taking the final diagnosis as the gold standard, the accuracy of the two methods is analyzed for diagnosing aneurysms, and the specific results are plotted into graphs, as shown in Table 3 and Figure 4.

Aneurysms were divided into three groups according to their maximum diameter: small aneurysm group (maximum diameter <5 mm), middle aneurysm group (5 mm < maximum diameter <15 mm), and large aneurysm group (maximum diameter >15 mm). The average accuracy of 3D-CTA diagnosis based on virtual reality is 90.81%. Among them, the small aneurysm group has the lowest diagnosis accuracy, followed by the middle aneurysm group, and the large aneurysm has the best diagnosis effect; the average diagnosis accuracy of DSA is 73.86%. 3D-CTA based on virtual reality can observe the three-dimensional structure of the aneurysm from any angle in space and has a good display ability of the spatial relationship between the tumor-bearing artery, aneurysm, and the surrounding blood vessels and bony structures.

### 4.2. System Application and Feedback

(1) The surgical path of the surgical treatment is planned through virtual reality-based 3D-CTA. Intracranial tumors are mainly performed by understanding the size, volume, location of the tumor, the blood supply artery and draining vein of the tumor, whether the skull is eroded, and evaluation and surgical approach planning. Twelve patients with the same symptoms and conditions were selected for microsurgery treatment, and they were divided into two groups with 6 people in each group. All patients in the experimental group used virtual reality-based 3D-CTA-related systems for diagnosis and surgical planning and treatment, while patients in the control group used DSA for diagnosis and surgical planning and treatment.
  1. The operation time of the two methods is shown in Table 4 and Figure 5.
  2. The human brain is the most complex part of the human anatomical structure. The brain is the commander of the human body. The brain contains various blood vessels, nerves, and functional areas that are extremely important to the human body to control the human body's language, movement, emotion, memory, cognition, etc. It has a series of advanced functions of the human body; therefore, there are great risks and uncertainties in the surgical treatment of intracranial lesions, which are truly affecting the whole body. Because blood vessels, nerves, and functional areas in the brain are easily damaged during surgery, the size, volume, and anatomical relationship between the surrounding blood vessels, nerves, skull, and adjacent important structures are detailed before neurosurgery. Understanding is very necessary and a prerequisite for the success of the operation.
  3. The comparison of the two diagnosis methods and the complications of the patients after treatment is shown in Table 5 and Figure 6.
  4. With the development of computer image processing technology, medical imaging technology, virtual reality, and other technologies, medical three-dimensional visualization technology has emerged and is widely used. The three-dimensional visualization technology of medical images is a technology that uses two-dimensional tomographic images scanned by traditional CT, MRI, etc. to reconstruct a three-dimensional model and perform qualitative and quantitative analysis of lesions. Three-dimensional visualization is also called three-dimensional reconstruction. The three-dimensional reconstruction of medical images is to use the visual characteristics of humans to transform human organs or lesions into images with three-dimensional effects through computer image processing technology, computer graphics, and human-computer interaction technology. Because the medical three-dimensional reconstruction technology has unmatched advantages in medical teaching, disease diagnosis, and treatment, it is widely concerned and highly praised by the medical community.
(2) After the doctor adopts the application system based on 3D-CTA virtual reality technology in intracranial aneurysm surgery to diagnose and treat the patient, we conduct a face-to-face interview to investigate the feedback situation used by 10 doctors, calculate the results, and organize and draw graphs, as shown in Table 6 and Figure 7.

It can be seen from the interview results that the vast majority of doctors agree with the application system based on 3D-CTA virtual reality technology in intracranial aneurysm surgery, accounting for 90%; most doctors believe that the application of this virtual reality operating system can promote confidence in treating patients, accounting for 80%.

## 5. Conclusions

At present, traditional surgical training has great limitations. With the rapid development of computer technology and virtual reality technology, a virtual surgical system combined with modern medical technology has emerged. The virtual surgery system can not only improve the efficiency and effectiveness of surgery learning and training to a large extent but also perform preoperative planning and rehearsal of rare operations. This paper studies the application of virtual reality technology to 3D-CTA intracranial aneurysm surgery, proposes the signal preprocessing algorithm and force feedback Euler algorithm in the virtual reality system, and designs the 3D-CTA virtual reality technology for intracranial aneurysm application system in surgery. The shortcomings of this article are that the number of experiments is not enough, and the experimental equipment is relatively backward, resulting in inaccurate results, which will be more in-depth in future research.

## Figures and Tables

**Figure 1:** Intracranial three-dimensional CT angiography.

**Figure 2:** Part of the technical process of the method in this article.

**Figure 3:** Execution time (s).

**Figure 4:** The correct rate of diagnosis of aneurysms of different sizes by 3D-CTA and DSA.

**Figure 5:** Operation time of 3D-CTA and DSA (min).

**Figure 6:** Comparison of complications (number of people).

**Figure 7:** Doctor's feedback.

**Table 1:** Some steps of the experiment in this article.

Application system design of intracranial aneurysm surgery based on 3D-CTA virtual reality technology	3.1	Overall system design	1	Human-computer interaction design
			2	Development tools
	3.2	Head posture tracking technology	1	VTK coordinate system
			2	Head posture acquisition method
			3	Display under threshold control

**Table 2:** Execution time (*s*).

Experiment number	Traditional Euler algorithm	Improved Euler algorithm	Runge-Kutta algorithm
1	12.37	4.29	16.73
2	14.48	5.31	18.21
3	15.69	5.94	17.42
4	13.07	6.15	15.89
5	16.27	5.03	16.35
6	15.47	4.84	18.56
Average	14.56	5.26	17.19

**Table 3:** The diagnostic accuracy of 3D-CTA and DSA for different sizes of aneurysms.

Aneurysm diameter	3D-CTA (%)	DSA (%)
Small aneurysm	86.71	67.42
Middle aneurysm	91.47	74.61
Large aneurysm group	94.25	79.54
Average	90.81	73.86

**Table 4:** Operation time of 3D-CTA and DSA (min).

Patient ID	3D-CTA	DSA
1	261.41	266.15
2	253.26	272.43
3	240.17	274.84
4	246.74	263.27
5	250.35	259.87
6	244.83	265.46

**Table 5:** Comparison of complications (number of people).

Complication	3D-CTA	DSA
Lung infection	2	4
Cerebrospinal fluid leakage	1	2
Intracranial hemorrhage	1	3
Epilepsy	3	2
Neurological dysfunction	2	3
Intracranial infection	1	1

**Table 6:** Feedback from doctors.

Serial number	Interview content	Yes	Yes percentage (%)	No	No percentage (%)
1	Do you like the application system based on 3D-CTA virtual reality technology in intracranial aneurysm surgery?	9	90	1	10
2	Does this application system help you improve your medical skills?	7	70	3	30
3	Does this application system help you increase your confidence in surgery?	6	60	4	40
4	Does this application system make you feel convenient?	8	80	2	20
5	Is this application system smart?	10	100	0	0

## Data Availability

Data sharing is not applicable to this article as no datasets were generated or analyzed during the current study.
